The article "Video Image Moving Target Recognition Method Based on Generated Countermeasure Network" was published in 2022. Journal: Comput Intell Neurosci.

# Video Image Moving Target Recognition Method Based on Generated Countermeasure Network

**DOI:** 10.1155/2022/7972845

**Published:** 2022-08-19

**Authors:** Zilong Li, DaiHong Jiang, Hongdong Wang, Dan Li

**Affiliations:** ^1^School of Information Engineering, Xuzhou University of Technology, Xuzhou 221018, China; ^2^School of Computer Science & Technology, China University of Mining and Technology, Xuzhou 221116, China; ^3^Post-Doctoral Research Center, Onnes Power Technology Co.Ltd., Xuzhou 221003, China

## Abstract

In order to improve the accuracy of video image moving target recognition and shorten the recognition time, a video image moving target recognition method based on a generation countermeasure network is proposed. Firstly, the image sensor is used to collect the video image and obtain the video image sequence. The Roberts operator is used for edge detection and Gaussian smoothing of the video image. Secondly, the normalization method is used to extract the key features of moving targets in video images. Finally, training is carried out alternately to generate the countermeasure network model, and the video image moving target recognition sample results are output according to the training results to realize the video image moving target recognition. The experimental results show that the highest recognition accuracy of the proposed method is 98.1%, and the longest recognition time is only 5.7 s, indicating that its recognition effect is good.

## 1. Introduction

Vision is the most direct way for people to get information. Images are the main way for humans to visually obtain information, and images can vividly and vividly describe the dynamic state of images and can convey information more intuitively and specifically [1–3]. With the advancement of science and technology, the development of computer vision technology has gradually made up for and improved the ability of people's vision that they do not have. Among these data, images and videos are important information carriers for computer vision systems. Recognition of moving objects is the key technology of visual analysis of moving objects, and it is also the most basic problem. It usually extracts moving images from the background and preprocesses them [4–6]. When performing target recognition, it is necessary to effectively detect the target and to classify and preprocess it to facilitate subsequent processing. In each frame of video, each independent moving object or region of interest to the user can be quickly and accurately identified and positioned to the next node. Therefore, it is of great significance to identify moving objects in video images.

At present, scholars in related fields are studying the recognition of moving objects in video images. Reference [7] proposed a video moving object recognition method based on hierarchical modeling and alternating optimization. Based on the observation that foreground and background are two sides of the same coin, treat them as equivalent unknown variables and pose a joint estimation problem called hierarchical modeling and alternating optimization. For the background, it is decomposed into low and high frequency components in time. For the foreground, a Markov random field is constructed as the axis at low spatial resolution. Based on the hierarchical extension of the two models, under a unified framework called the alternating direction multiplier method, the joint estimation is improved to realize video moving target detection and recognition. Experimental results show that this method can generate more discriminative backgrounds and has better robustness to noise, but there is a problem of low recognition accuracy. Reference [8] proposed a moving target recognition method in a high dynamic scene of a visual prosthesis. A new unsupervised moving target segmentation model is constructed to automatically extract moving targets in high dynamic scenes. The model utilizes foreground cues with spatiotemporal edge features and background cues with boundary priors to generate proximity maps of moving objects in dynamic scenes according to a manifold ranking function. At the same time, foreground and background cues are ranked, and moving objects are extracted through the integration of the two ranking maps. Experimental results show that this method can evenly highlight moving objects in high dynamic scenes and maintain a good boundary, but there is a problem of long recognition time. Reference [9] proposed a moving target recognition method based on sparse and robust principal component analysis of spatiotemporal structure in complex scenes. The algorithm spatially and temporally regularizes the sparse components in the form of the graph Laplacian. Each Laplacian corresponds to a multifeature map constructed over superpixels in the input matrix. The sparse components are used as eigenvectors for the spatial and temporal graph Laplacian while minimizing the robust PCA objective function. A novel objective function is obtained for separating moving objects in complex backgrounds. The proposed objective function is solved using a linear alternating directions method with multiplier-based batch optimization. In addition, an online optimization algorithm for real-time applications is also proposed. Batch and online solutions are evaluated using six publicly available datasets containing most of the above-given challenges. The experimental results show that the algorithm has higher performance, but there is a problem of poor recognition effect.

In order to solve the problems of low recognition accuracy of video images, long recognition time, and poor recognition improvement in traditional methods, this paper proposes a video image moving target recognition method based on a generative adversarial network. The specific technical route studied in this paper is as follows:

  Step 1: collect a real-time image through an image sensor to obtain a video image sequence, preprocess the collected video image sequence, use the Roberts operator to perform edge detection on the video image, and perform Gaussian smoothing on the video image at the same time
  Step 2: according to the video image preprocessing result, after the feature vector of the video image moving target is obtained by using the normalization processing method, the key features of the video image moving target are extracted
  Step 3: train the generative adversarial network model through interactive training, identify the video image moving target according to the training result and the key features of the moving target, and output the moving target recognition sample, thereby realizing the video image moving target recognition
  Step 4: comparing the proposed method with the method of reference [7] and the method of reference [8], the experimental results and conclusions are drawn

## 2. Design of Video Image Moving Target Recognition Method

### 2.1. Video Image Preprocessing

The object of video image moving target recognition is video image sequence, which is also called video sequence and dynamic image [10, 11]. A video image sequence is a series of video images with a certain or assumed relative order acquired by an image sensor, and the time interval between two adjacent two pictures is given. The video image sequence can generally be expressed as follows:

(1) $$\begin{array}{c} Q=\left\{q\left(e,r,w_{0},e,r,w_{1},\ldots ,e,r,w_{N-1}\right)\right\}. \end{array}$$

Or,

(2) $$\begin{array}{c} Q={\left\{q_{k}\left(e,r\right)\right\}}_{k=1}^{N}. \end{array}$$

In formulas (1) and (2), *w*_*i*_, *i*=0,1,…, *N* − 1 is the moment when the frame of video image is acquired, *e*, *r* is the direction of the sensor in the imaging interval, *k* is the frame sequence, and *N* is the total number of frames of the video image sequence.

Due to the restriction of the acquisition environment and the influence of random interference and other factors, the effect of recognizing the moving target of the video image is not good, and it needs to be preprocessed. It consists of two steps: edge detection and smooth noise reduction.

#### 2.1.1. Video Image Edge Detection

There are many operators for edge detection, and the fixed template is convolved to obtain the edge of the image. Select Roberts operator [12] to complete video image edge detection.

The video image gradient and the first-order derivative operator correspond to each other. Assuming that the video image function is expressed as *Q*(*u*, *o*), its gradient is defined as follows:

(3) $$\begin{array}{c} \nabla Q\left(u,o\right)=\left(U_{u},U_{o}\right)=\left(\frac{\alpha u-\alpha o}{\alpha u+\alpha o}\right). \end{array}$$

In formula (3), *U*_*u*_ and *U*_*o*_ represent the gradients at pixels *u* and *o* of the video image, respectively, and *α* is a vector factor. Then, the magnitude of this vector is as follows:

(4) $$\begin{array}{c} \beta =\left|\nabla Q\left(u,o\right)\right|=\frac{U_{u}^{2}}{U_{o}^{2}}. \end{array}$$

For ease of calculation, the magnitude can be expressed in the following different ways:

(5) $$\begin{array}{c} \left\{\begin{array}{c} \beta =\max\left(U_{u},U_{o}\right)\\ \beta =\left|U_{u}\right|+\left|U_{o}\right| \end{array}\right.. \end{array}$$

Using Roberts operator, the process of realizing video image edge detection is described as follows:

(6) $$\begin{array}{c} Y\left(u,o\right)=\beta \left[P\left(u,o\right)-P\left(u+1,o+1\right)+P\left(u+1,o\right)\right]. \end{array}$$

In formula (6), *Y*(*u*, *o*) and *P*(*u*, *o*)_,_ respectively, represent the gray value of the pixel point (*u*, *o*) before and after the edge detection of the video image.

#### 2.1.2. Gaussian Smoothing of Video Image

In the process of edge detection, the noise will cause the edge contour curve of the video image to be not smooth enough, which reduces the description accuracy of the edge contour curve of the video image. To this end, for video images, Gaussian smoothing is also required [13–15]. Assuming that the contour curve of the video image is represented as *A*, and *A*(*i*) is the set of all pixels on the contour curve of the video image, there are

(7) $$\begin{array}{c} A=\left\{A\left(i\right)=\left(u\left(i\right),o\left(i\right)\right)\right\}. \end{array}$$

In formula (7), *u*(*i*), *o*(*i*)_,_ respectively, represents the pixel points on the contour curve of the video image after Gaussian smoothing.

Using formula (7), all pixels in the outline of the video image can be traversed to achieve smoothing. After edge detection and smoothing, the video image quality is improved.

### 2.2. Extraction of Key Features of Moving Objects in Video Images

Based on the video image preprocessing results, the key features of moving objects are extracted. In order to improve the accuracy of video image moving target recognition, after normalizing the video image moving target feature vector, the key features of the video image moving target are extracted. The normalization processing method does not require geometric correction of moving objects in video images and can achieve a higher feature recognition rate, reduce the complexity of key feature extraction of objects, and basically eliminate the influence of changes in moving objects in images on feature extraction results., with high application value.

(1) Normalization of video image moving target feature vector [16, 17]: the depth value of a video image moving target pixel and its neighboring pixels is regarded as the video image moving target feature. Then, the feature vector expression of the video image moving target is as follows:
  (8) $$\begin{array}{c} S\left(u,o\right)=\frac{\left[D\left(u-1,o-1\right),D\left(1-u,1-o\right)\right]}{\left[D\left(u,o+1\right),D\left(u+1,o\right)\right]}. \end{array}$$
In formula (8), *D*(*u*, *o*) is the depth value of the pixel point (*u*, *o*) of the video image. Perform the following normalization processing on all video image moving target feature vectors:
  (9) $$\begin{array}{c} S{\;}^{\prime }\left(u,o\right)=\frac{S\left(u,o\right)}{S\left(u,o\right)}. \end{array}$$
In formula (9), *S* ′(*u*, *o*) represents the normalized video image moving target feature vector.
After the above-given processing, the key parts of the video image are effectively preserved, thereby reducing the complexity of feature extraction for moving objects in the video image.
(2) Extraction of key features of moving objects in video images: after the feature vector of moving objects in video images is normalized, redundant features in moving objects in video images are removed. According to the shape of the moving target area of the video image, the key feature points of the moving target of the video image are determined, and the key lines are drawn from this point as the center. The specific operation process is described by the following formula:

(10) $$\begin{array}{c} \gamma =\overset{F}{\underset{n=5}{\prod }}\left[\frac{g_{n}-g_{1}}{\sqrt{{\left(g_{n}-g_{1}\right)}^{2}+\left(g_{n}-g_{1}\right)}}\right]+{\left|\frac{g_{n-1}-g_{1}}{\sqrt{{\left(g_{n-1}-g_{1}\right)}^{2}+\left(g_{n-1}-g_{1}\right)}}\right|}^{2}. \end{array}$$

In formula (10), *g*_*n*_ represents the image moving target key point, *n* is the number of video image moving target key points, and *F* is the video image moving target key feature point set. After the above process, the key features of the video image moving target are effectively extracted, which lays a foundation for the video image moving target recognition.

### 2.3. Realization of Video Image Moving Target Recognition

The establishment of a generative adversarial network is based on game theory, which includes two aspects, namely, the generative model and the discriminative model [18–20]. By establishing a generative adversarial network model, using the interactive training generative adversarial network model, optimizing the discriminant network and the generator network, and outputting the video image moving target recognition sample results, the video image moving target recognition is realized. Compared with traditional methods, the generative adversarial network has the following advantages: in principle, the generative adversarial network can approach any probability distribution gradually and can be considered as a nonparametric production modeling method. If the discriminator is well trained, the generator can learn the distribution of training samples perfectly. In the generation countermeasure network training, the reconstruction loss weighting coefficient is set to 0.999, and the countermeasure loss weighting coefficient is set to 0.001.

The objective function of the generative adversarial network model used to realize the recognition of moving objects in video images is derived as follows:

(11) $$\begin{array}{c} \underset{L}{\min}\underset{K}{\max}J\left(K,L\right)=Z_{x∼c_{d}\left(x\right)}\times \left[\mathrm{lg}\left(K\left(x\right)\right)\right]+Z_{h∼c_{h}\left(h\right)}\times \left[\mathrm{lg}\left(1-K\left(L\left(h\right)\right.\right)\right]. \end{array}$$

In formula (11), *x* is the video image, *J*(*K*, *L*) is the generative adversarial network model function, and *K*, *L* is the discriminative model and the generative model. *Z*_*x*∼*c*_*d*_(*x*)_ refers to the expected value of the actual data after passing through the discriminator, *x* ~ *c*_*d*_(*x*) means that *x* is subject to the actual data distribution, and *K*(*x*) is the discriminator. *Z*_*h*∼*c*_*h*_(*h*)_ refers to the expected value of random data after the generator and discriminator, *h* ~ *c*_*h*_(*h*) refers to the sampling distribution of the randomly generated video image moving objects, and *L*(*h*) refers to the generator.

In the training of the discriminator network and the generator network, the alternate training method is adopted, which is optimized, and the corresponding training steps are given:

Step 1: pretrain the generative adversarial network initial discriminator network.
Step 2: input the moving target of the video image to be trained into the discriminator network to obtain the mask *δ*.
Step 3: extract *ε* moving target samples from training real video images and their corresponding masks *δ*_*ε*_. Input *ε* real video image moving target samples into the discriminator. Input the *ε* real video image moving target samples and the corresponding mask *δ*_*ε*_ into the generator, generate the realistic video image moving target samples, and input the realistic video image moving target samples into the discriminator.
Step 4: calculate the discriminator loss function according to the discriminant situation:
  (12) $$\begin{array}{c} G^{D}=\frac{1}{\varepsilon }\left[-\mathrm{lg}\left(K\left(x\right)\right)-\mathrm{lg}\left(1-K\left(L\left(h,\delta_{\varepsilon }\right)\right)\right)\right]. \end{array}$$
Step 5: the discriminator network parameters are updated by the Adam gradient descent algorithm:
  (13) $$\begin{array}{c} \theta_{d}=\text{Adam}\left(\delta_{\varepsilon }\left(G^{D}\right),\theta_{d}\right). \end{array}$$
Step 6: according to the discriminant situation, calculate the generator loss function:
  (14) $$\begin{array}{c} G^{H}=\frac{1}{\varepsilon }\left[\mathrm{lg}\left(1-K\left(L\left(h,\delta_{\varepsilon }\right)\right)\right)\right]. \end{array}$$
Step 7: the generator network parameters are updated by the Adam gradient descent algorithm:
  (15) $$\begin{array}{c} \theta_{h}=\text{Adam}\left(\delta_{\varepsilon }\left(G^{H}\right),\theta_{d}\right). \end{array}$$
Step 8: repeat step 3 until the upper limit of the number of iterations or the generative adversarial network is close to the Nash equilibrium, and the result of the output video image moving target recognition sample is:

(16) $$\begin{array}{c} \mu =\left(G^{D}\times \theta_{d}\right)-\left(G^{H}\times \theta_{h}\right). \end{array}$$

According to the above-given analysis, the method in this paper first collects the video image through the image sensor and uses the Roberts operator to preprocess the video image to obtain the results of edge detection and Gaussian smoothing. On this basis, the key features of moving objects in video images are obtained by normalized processing, and the recognition of moving objects in video images is realized by using the generative adversarial network to output the sample results of moving objects in video images.

Through the above-given process, the recognition of moving objects in video images based on the generative adversarial network is realized.

## 3. Experimental Analysis

### 3.1. Experimental Design

In order to verify the effectiveness of the video image moving target recognition method based on a generative adversarial network, experimental tests are carried out.

1. Experimental hardware environment: the experimental test platform is 64 bit Ubuntu14.04, and the specific parameters of the platform are shown in Table 1.
2. Source of experimental data: the images used in this paper are all from the VOC2007 public dataset, which includes 20 different types of video images. Among them, including 5011 pictures and 4952 video images, 50 video image moving objects are selected from this dataset as experimental data to identify the video image moving objects. In order to improve the accuracy of the experimental results, it is necessary to ensure the consistency of the image sample specifications used in the experiment, and to process the samples through MATLAB software.
3. Experimental indicators: in the experiment, the video image moving target recognition effect, recognition accuracy, recognition time, target recognition quantity, and recognition rate are analyzed as performance indicators.
4. In the experiment, the method of reference [7], the method of reference [8], and the proposed method were used to compare and verify the effectiveness of the proposed method.

### 3.2. Testing and Analysis of Performance Indicators

Two video images were selected for recognition in the experimental data set to verify the recognition effect of the proposed method on moving objects. By comparing the method of reference [7], the method of reference [8], and the proposed method, the recognition effects of different methods on moving objects in video images are obtained, as shown in Figure 1 and Figure 2.

According to Figure 1, it can be seen that the recognition result of the video image moving target obtained by the method of reference [7] is too dark, and the recognition effect is not good due to too much noise interference. The video image moving target recognition result obtained by the method of reference [8] is too bright, and the recognition effect is also poor because the edge is not clear enough. In addition, both methods are not good at identifying moving objects. However, the proposed method recognizes moving objects and obtains good results, with moderate brightness, low noise, and clear edges of moving objects. It can be seen from this point that the proposed method is effective and the recognition effect is better.

It can be seen from Figure 2 that when the proposed method is used to identify the moving target in image 2, the head, hands, legs, and footsteps of the athlete in the image can be effectively identified, and the movements are independent of each other and do not appear to identify problems with confusing results. In the recognition method of reference [7], some head movements and footsteps are missing, and the recognition results are not comprehensive enough. The method of reference [8] has the problem of confusion in recognition and recognizes the actions of different moving subjects as one part. It can be seen from the above analysis that the proposed method has a better recognition effect.

To further verify the accuracy of the video image moving target recognition of the proposed method, the method of reference [7], the method of reference [8], and the proposed method are used to compare, and the accuracy of video image moving target recognition of different methods is shown in Figure 3.

According to Figure 3(a), it can be seen that the difference between the recognition accuracy of video images of the three methods is small. The recognition accuracy of the proposed method is compared with the method in reference [7] and reference [8]. There are certain advantages, but the advantages are not obvious.

According to Figure 3(b), when there are 50 moving objects in the video image, the average video image moving target recognition accuracy of the method of reference [7] is 82.9%, and the average video image moving target recognition accuracy of the method of reference [8] is 66.2%. The average video image moving target recognition accuracy of the proposed method is as high as 98.1%. It can be seen that the proposed method has a high accuracy of video image moving target recognition. This is because the proposed method uses the normalization processing method to extract the moving target features of the video image. This method does not require geometric correction of the moving target in the video image but also achieves a high feature recognition rate and reduces the time required for the extraction of key features of the target. Complexity, which is beneficial to improve the accuracy of target recognition.

On this basis, the proposed method is further verified for the recognition time of moving objects in video images. Comparing the method of reference [7] and the method of reference [8] with the proposed method, the recognition time of moving objects of different methods is obtained, as shown in Table 2.

According to Table 2, with the increase of moving objects in video images, the recognition time of moving objects in video images by different methods increases. When there are 50 moving objects in the video image, the recognition time of the method of reference [7] is 12.5 s, and that in the method of reference [8] is 14.4 s. The time for the proposed method to recognize moving objects in video images is only 5.7 s. It can be seen that the proposed method has a short time for the recognition of moving objects in video images. This is because the proposed method preprocesses the video image before target recognition, which is conducive to more efficient target recognition.

There may be a large number of moving targets in the video image, and whether these targets can be comprehensively recognized is also a key indicator to verify the proposed method. Comparing reference [7] method and reference [8] method with the proposed method, the number of moving targets recognized by different methods is obtained, and the results are shown in Table 3.

It can be seen from the data in Table 3 that when the proposed method is used for target recognition on 10 video images, the number of recognized targets is significantly higher than that of reference [7] method and reference [8] method. Taking image 5 as an example, the proposed method identified 31 targets, reference [7] method identified 25 targets, and reference [8] method identified 27 targets; taking image 8 as an example, the proposed method identified 27 targets, 22 targets were identified by reference [7] method, and 23 targets were identified by reference [8] method. By comparison, it can be seen that the number of targets identified by the proposed method is more, indicating that the identification results of this method are more comprehensive. This is because the method uses the normalization processing method to extract the key features of moving objects in video images, which is beneficial to improve the comprehensiveness of object recognition.

Finally, the target recognition rate is used as the experimental index to compare the moving target recognition effects of reference [7] method, reference [8] method, and the proposed method. The results are shown in Figure 4.

According to Figure 4, with the increase of the number of experiments, the recognition rate of reference [7] method, reference [8] method, and the proposed method shows a rapid upward trend, but the recognition rate of the proposed method is always higher than that of reference [7] method and reference [8] method. The highest recognition rate of the proposed method is 95%, which is increased by 11% and 13% respectively compared with reference [7] method and reference [8] method. It can be concluded that the recognition effect of the proposed method is better, which further verifies its application value.

## 4. Conclusion

In order to effectively improve the accuracy of video image moving target recognition, ensure the recognition effect, and shorten the recognition time, a method for video image moving target recognition based on the generative adversarial network is proposed. The main innovations of this method are as follows:

1. A video image acquisition method based on an image sensor is adopted to acquire a video image sequence.
2. Select the Roberts operator to detect the edge of the video image, use Gaussian smoothing, and then standardize it to obtain the key features of the moving target.
3. By establishing a generative adversarial network model, training it, optimizing the discriminant and generator networks respectively, and outputting the sample results of video image moving target recognition to realize video image moving target recognition.
4. The experimental results show that the proposed method has a good recognition effect, with moderate brightness, low noise, and clear moving target edges. The recognition accuracy rate reaches 98.1%, and the recognition time is only 5.7 s.

## Figures and Tables

**Figure 1:** Image 1 recognition effect. (a) The proposed method. (b) Reference [7] method. (c) Reference [8] method.

**Figure 2:** Image 2 recognition effect. (a) The proposed method. (b) Reference [7] method. (c) Reference [8] method.

**Figure 3:** Video image moving target recognition accuracy of different methods. (a) Unobstructed. (b) Partial occlusion.

**Figure 4:** Comparison results of recognition rates of different methods.

**Table 1:** Parameter settings of the experimental test platform.

Name	Specific parameters
CPU	i7-6770K@4.00 GHz
Hard disk	1 TB SSD
Graphics card	AMD
Memory	8G
Operating system	Windows 10

**Table 2:** Video image moving target recognition time by different methods.

Video image moving target (piece)	The proposed method (s)	The method of reference [7] (s)	The method of reference [8] (s)
10	1.2	4.1	6.5
20	2.5	6.8	8.3
30	3.6	8.6	10.8
40	4.8	10.3	12.7
50	5.7	12.5	14.4
60	6.0	13.1	15.4
70	6.5	14.6	16.3
80	6.9	15.2	17.0
90	7.2	16.7	17.6
100	7.4	17.9	18.3

**Table 3:** Comparison results of target recognition number of different methods.

Video image number	The proposed method	The method of reference [7]	The method of reference [8]
1	35	27	34
2	41	38	36
3	29	26	26
4	24	21	19
5	31	25	27
6	34	30	30
7	40	34	35
8	27	22	23
9	26	23	20
10	33	28	28

## Data Availability

The data used to support the findings of this study are available from the corresponding author upon request.
